The article "SPARC Overexpression Inhibits Cell Proliferation in Neuroblastoma and Is Partly Mediated by Tumor Suppressor Protein PTEN and AKT" was retracted in 2020. Reasons: fabricated or falsified data; an official misconduct investigation; misconduct by an author; duplicated images.

# SPARC Overexpression Inhibits Cell Proliferation in Neuroblastoma and Is Partly Mediated by Tumor Suppressor Protein PTEN and AKT

**DOI:** 10.1371/journal.pone.0036093

**Published:** 2012-05-02

**Authors:** Praveen Bhoopathi, Bharathi Gorantla, G. S. Sailaja, Christopher S. Gondi, Meena Gujrati, Jeffrey D. Klopfenstein, Jasti S. Rao

**Affiliations:** 1 Department of Cancer Biology and Pharmacology, University of Illinois College of Medicine at Peoria, Peoria, Illinois, United States of America; 2 Department of Pathology, University of Illinois College of Medicine at Peoria, Peoria, Illinois, United States of America; 3 Department of Neurosurgery, University of Illinois College of Medicine at Peoria, Peoria, Illinois, United States of America; Sun Yat-sen University Medical School, China

## Abstract

Secreted protein acidic and rich in cysteine (SPARC) is also known as BM-40 or Osteonectin, a multi-functional protein modulating cell–cell and cell–matrix interactions. In cancer, SPARC is not only linked with a highly aggressive phenotype, but it also acts as a tumor suppressor. In the present study, we sought to characterize the function of SPARC and its role in sensitizing neuroblastoma cells to radio-therapy. SPARC overexpression in neuroblastoma cells inhibited cell proliferation *in vitro*. Additionally, SPARC overexpression significantly suppressed the activity of AKT and this suppression was accompanied by an increase in the tumor suppressor protein PTEN both *in vitro* and *in vivo*. Restoration of neuroblastoma cell radio-sensitivity was achieved by overexpression of SPARC in neuroblastoma cells *in vitro* and *in vivo*. To confirm the role of the AKT in proliferation inhibited by SPARC overexpression, we transfected neuroblastoma cells with a plasmid vector carrying myr-AKT. Myr-AKT overexpression reversed SPARC-mediated PTEN and increased proliferation of neuroblastoma cells *in vitro*. PTEN overexpression in parallel with SPARC siRNA resulted in decreased AKT phosphorylation and proliferation *in vitro*. Taken together, these results establish SPARC as an effector of AKT-PTEN-mediated inhibition of proliferation in neuroblastoma *in vitro* and *in vivo*.

## Introduction

Neuroblastoma is the most common extracranial solid tumor in children under the age of five years. When neuroblastoma is first diagnosed, 50 percent of the patients are considered to be high-risk patients. Neuroblastoma originates from neural crest cells and these tumors, which are normally dissimilar both clinically and biologically, are found in the adrenal medulla or near the sympathetic chain [1]. Neuroblastoma in infants may regress spontaneously while tumors in older patients may settle into benign ganglioneuromas. Neuroblastoma is caused by rapid cell production by the neuroblast during fetal growth, which causes a growth or a tumor to develop. Usually, these tumors cannot be removed completely through surgery due to metastasis at the time of diagnosis and have a very poor prognosis. Metastasis is a complex process mainly dependent on cell adhesion to the extracellular matrix (ECM) and basement membrane and takes place through a multi-step process that includes cell infiltration from the primary tumor, intravascular invasion, and eventually proliferation to the metastatic site [2], [3] Although intensive multimodality therapies have produced some developments in the overall cure rate of these tumors, the therapies have considerable short- and long-term toxicities. Thus, a detailed knowledge of mechanisms controlling proliferation and differentiation may lead to a better understanding of the molecular pathogenesis of neuroblastoma, which may result in novel biologically-based therapies that are less toxic and more effective.

While the ECM is classically thought to instruct cell behavior primarily through biochemical recognition by cell adhesion receptors, signals encoded in the ECM may play a significant role in guiding neuroblastoma differentiation and proliferation. Overall, the mechanical stringency of the ECM can intensely alter cellular behavior, including morphology, motility, and proliferation [4]–[6]. The matricellular proteins are extracellular proteins and do not contribute structurally to the extracellular environment as do the classical extracellular matrix proteins, but instead they modulate interactions between the extracellular matrix and cells. One such matricellular protein is Secreted Protein Acidic and Rich in Cysteine (SPARC), also known as osteonectin or BM-40, a 34 kDa, calcium-binding glycoprotein shown to associate with the cell membrane and membrane receptors [7], [8]. SPARC is known to not only modulate cell–cell and cell–matrix interactions, but also to influence de-adhesive and growth regulatory properties [9]. In cancers, SPARC may elicit different actions, showing the complexity of the protein [10], [11]. In certain types of cancers, like melanomas and gliomas, SPARC is associated with a highly aggressive tumor phenotype [9], whereas in other cancers, mainly ovarian, neuroblastomas, colorectal and PNET tumors, SPARC may function as a tumor suppressor [9], [12]. Recent studies show that SPARC modulates cellular functions and proliferation through modulation of different growth factor signaling [13]. In addition, we have shown that SPARC inhibits medulloblastoma tumor growth both *in vitro* and *in vivo* by inducing autophagy-mediated cell death and causing neuronal differentiation [14].

The tumor suppressor phosphatase and tensin homolog deleted on chromosome 10 (PTEN) is a phosphatase, which is deleted or mutated in a variety of human cancers [15]–[17]. PTEN plays an important role in keeping the processes of cell migration and proliferation under control. PTEN is a negative regulator of phosphatidylinositol-3-kinase (PI3K) signaling by dephosphorylating phosphatidylinositol- 3–5-triphosphate (PIP3). However, very little is known about the existence of other substrates for PTEN, with the exception of PtdIns-3,4,5-P3 and PtdIns-3,4-P2, which are required for the phosphorylation and activation of the AKT protein kinase, a survival factor that fuels the progression of the cell cycle [18]–[20] and also prevents cells from undergoing apoptosis by inhibiting pro-apoptotic factors as well as nuclear translocation of the forkhead transcription factors [21]–[23].

Earlier studies from our laboratory and others have shown that high levels of SPARC correlate with inhibited proliferation in many cancer types. We have shown that SPARC overexpression by an adenoviral vector induced autophagy-mediated apoptosis in PNET tumor cells. In the present study, we sought to further characterize the mechanism by which SPARC is capable of inhibiting proliferation in neuroblastoma cells.

## Results

### Overexpression of SPARC in neuroblastoma cells *in vitro*

SPARC, a prototype of the matricellular protein family, has been shown to play an important role in various aspects of tumorigenesis including tumor invasion, angiogenesis and tumor growth [12]. To elucidate the effect of SPARC overexpression using a genetic approach and to observe its effects on neuroblastoma tumor growth *in vitro* and *in vivo*, we subcloned a human SPARC cDNA in a pcDNA3.1 mammalian expression vector and transfected it into SK-N-AS, NB-1691 and IMR-32 neuroblastoma cells. Figure S1A shows that SPARC protein levels were increased in the three cell lines when compared to mock or empty vector-transfected cells. We observed a ∼3- to 4-fold increase in SPARC protein levels in pSPARC-transfected cells compared to controls. To confirm that this upregulation of SPARC mRNA translated into increased levels of SPARC protein, we assessed mRNA transcript levels in the pSPARC-transfected cells. SPARC-overexpressed neuroblastoma cells showed a 3- to 4-fold increase in mRNA levels when compared to mock or empty vector-transfected cells (Fig. S1B). As assessed by immunofluorescence microscopy, intense staining for SPARC was observed in all three cell lines transfected with pSPARC when compared to mock or empty vector-transfected cells (Fig. S1C). We compared the SPARC levels in tumor cells with HMEC cells (as control cells) and did not find much change in SPARC levels (Fig. S1D).

### X-ray radiation inhibits SPARC expression in neuroblastoma cells

SPARC has been shown to be a therapy-resistant reversal gene whose expression was significantly decreased in resistant cancer cells [24]. To determine whether there was a dose-dependent radiation effect on these cells we performed an *in vitro* clonogenic assay to characterize the survival of neuroblastoma cells, after exposure to ionizing radiation. SK-N-AS, NB1691 and IMR-32 cells were given a single dose of radiation (from 2 Gy to 12 Gy) and assayed for survival. Irradiated cells showed a dose-dependent decrease in survival fraction with a 27.6% survival rate at 8 Gy for SK-N-AS, a 30% survival rate at 8 Gy for NB1691 and a 25% survival rate at 4 Gy for IMR-32 cells when compared to non-radiated cells (Fig. S1E). To examine the effect of radiation on SPARC expression, we determined SPARC protein levels in SK-N-AS, NB1691 and IMR-32 neuroblastoma cells. Figure 1A indicates that SPARC expression levels were inhibited with radiation in a dose-dependent manner when compared to non-irradiated cells. Densitometric analysis revealed about 30–40% inhibition in SPARC levels when cells were treated with 8 Gy (SK-N-AS and NB1691) and 4 Gy in IMR-32 cells as compared to non-irradiated cells.

**Figure 1:** Irradiation inhibits SPARC expression and inhibits proliferation of neuroblastoma cells. (**A**) SK-N-AS, NB1691 and IMR-32 cells were irradiated (IR) with X-ray (0–12 Gy), incubated for 12 hours, and cells were collected. (A) SPARC expression was determined by western blot analysis in cell lysates. Results are representative of three independent experiments. GAPDH served as a loading control. Columns, mean of three experiments; bars, SD. (**B**) Neuroblastoma cell lines SK-N-AS, NB1691 and IMR-32 cells were transfected with mock (PBS control), empty vector (pEV) or pSPARC for 24 hours, and SK-N-AS and NB1691cells were irradiated with 8 Gy and IMR-32 cells were irradiated with 4 Gy dose of radiation. ***Left panel*** **:** SPARC levels were determined by Western blot analysis using a SPARC-specific antibody. GAPDH served as a loading control. ***Middle panel*** **:** cDNA was produced from total RNA extracted from the mock and infected cells. RT-PCR was performed for SPARC. Results are representative of three independent experiments. GAPDH served as a control for RNA quality. ***Right panel*** **:** Densitometric analysis showing levels of SPARC protein and mRNA levels. Columns, mean of three experiments; bars, SD. * *p*<0.01 vs pEV; ** *p*<0.01 vs IR+pEV. (**C**) SK-N-AS, NB-1691 and IMR-32 cells were transfected with mock, pEV or pSPARC and at the indicated time points, the plates were incubated by adding MTT reagent for a further 6 hours. The developed purple color Formazan crystals were solubilized using DMSO, and color intensity was measured using a spectrophotometer at 570 nm. Data were plotted as absorbance at 570 nm. Results are representative of three independent experiments. Points, mean of three experiments. H = hours. (**D**) SK-N-AS, NB1691 and IMR-32 neuroblastoma cells were transfected with mock, pEV or pSPARC. After 24 hours of incubation, SK-N-AS and NB1691 cells were irradiated with 8 Gy; IMR-32 cells were irradiated with 4 Gy and clonogenic assay was performed as described in Materials and Methods. The cells were cultured and colonies larger than 50 cells were counted. Columns: mean of triplicate experiments; bars: SD. (**E**) SK-N-AS, NB1691 and IMR-32 neuroblastoma cells were transfected with mock, pEV or pSPARC. After 24 hours of incubation, SK-N-AS and NB1691 cells were irradiated with 8 Gy and cultured for another 16 hours. TUNEL assay was performed as per the manufacturer's procedure. (**F**) SK-N-AS neuroblastoma cells were transfected with mock, pEV or pSPARC. After 24 hours of incubation, cells were irradiated with 8 Gy and cultured for another 16 hours. Western blot analysis was performed for Caspase3 and PARP specific antibodies and GAPDH served as loading control.

### SPARC overexpression inhibits proliferation in neuroblastoma cells

We next examined the possible role of SPARC in radiation response. Inhibition of SPARC levels by radiation was restored using a plasmid vector encoding the SPARC full-length gene. SPARC overexpression in neuroblastoma cell lines prior to irradiation exhibited increased SPARC protein and transcript levels in neuroblastoma cell lines (Fig. 1B) when compared to mock or empty vector-treated cells prior to irradiation. Densitometric analysis for SPARC protein and transcript levels showed a 3- to 4-fold increase (Fig. 1B) in the pSPARC treatment prior to irradiation. Further, we assessed the sensitivity of neuroblastoma cells to SPARC overexpression in combination with radiation using the MTT proliferation assay. The results revealed that SPARC-overexpressed cells had increased sensitivity to radiation, and their proliferation rate was less than that of cells treated with radiation alone or combined with mock or empty vector treatment (Fig. 1C). We also assessed the impact of the combination treatment on neuroblastoma cells using clonogenic survival assay and found that combining SPARC and ionizing radiation resulted in increased cell death (Fig. 1D). To further confirm the effect of SPARC overexpression on neuroblastoma cell growth, we performed TUNEL assay. SPARC overexpression in neuroblastoma cell lines prior to irradiation exhibited increased TUNEL positive cells compared to that of cells treated with radiation alone or combined with mock or empty vector treatment (Fig1E). To further confirm this result, we also analyzed cleavage of PARP and caspase3 by western blot analysis. Western blot analysis revealed that SPARC overexpression in neuroblastoma cell line (SK-N-AS) prior to irradiation exhibited increased cleavage of capspase3 and PARP when compared to that of cells treated with radiation alone or combined with mock or empty vector treatment (Fig. 1F).

### SPARC overexpression abates irradiation-induced cell cycle arrest in neuroblastoma cells

When cells are exposed to radiation, they initiate a complex response that includes the arrest of cell cycle progression [25]. DNA is an important subcellular target of ionizing radiation, but oxidative damage to plasma membrane lipids initiates signal transduction pathways that activate apoptosis and may play a role in cell cycle regulation [26]. Moreover, irradiation-induced G2 arrest was shown to require inhibitory phosphorylation of the kinase Cdc2 [27]. To identify whether the growth inhibitory effect in cells that received the combined treatment of radiation and SPARC overexpression was caused by specific perturbation of cell cycle-related events, DNA contents of neuroblastoma cells were measured by flow cytometric analysis. Flow cytometric analyses using neuroblastoma cells treated with mock, empty vector (pEV), pSPARC with and without radiation (IR) demonstrated a significant increase in the proportion of G2/M cells and a reduced number of G1 cells after IR treatment when compared to controls. However, SPARC treatment prior to IR increased the number of sub-G1 cells as compared to SPARC treatment alone (Fig. 2A). As shown in Figure 2A, treatment of neuroblastoma cells with radiation resulted in an increase in the percentage of G2/M cells (from 10% to ∼50%) as compared to control, non-irradiated cells. In cells transfected with pSPARC prior to radiation, the percentage of cells in the sub-G1 phase increased to a maximum of 20%.

**Figure 2:** SPARC overexpression sensitizes neuroblastoma cells to radiation by abating irradiation-induced cell cycle arrest. SK-N-AS, NB1691 and IMR-32 cells were transfected with mock (PBS control), empty vector (pEV) or with pSPARC for 24 hours, and SK-N-AS and NB1691cells were irradiated (IR) with 8 Gy and IMR-32 cells were irradiated with 4 Gy dose of radiation. (**A**) Cells were collected and subjected to FACS analysis with propidium iodide staining for DNA content and represented in a graphical manner. Results are representative of three independent experiments. Columns: mean of triplicate experiments. (**B**) Cells were collected and the cell lysates were subjected to western blotting for Chk1, Chk2, Cdc25C, Cyclin B1, Cdc2 and pCdc2. Results are representative of three independent experiments. Densitometric analysis for Chk1 and Cdc25C is shown in the corresponding bar graph. Columns, mean of triplicate experiments; bars, SD. * *p*<0.01 vs pEV; ** *p*<0.01 vs IR+pEV.

Functional defect in DNA damage checkpoint pathways showed increased sensitivity to radiation and other DNA damage agents [28], [29]. This observation suggests a possibility that components of these DNA damage checkpoint pathways may serve as potential therapeutic targets for enhancing radiosensitivity of tumor cells [30]. To test this hypothesis, we evaluated the protein levels of Chk1 and phospho-Cdc25C in SPARC-overexpressed neuroblastoma cells. Irradiated neuroblastoma cell lines exhibited a significant increase in Chk1 levels but not in Chk2 levels. Further, irradiation-induced Chk1 levels were increased in cells treated with pSPARC prior to IR (Fig. 2B). Densitometric analysis for Chk1 and Cdc25C indicated 3- to 4-fold increase in SPARC-overexpressed cells when compared to mock or empty vector-treated cells (Fig. 2B). Recent studies showed that Chk1, a serine-threonine kinase, is critical for G2/M arrest in response to DNA damage and is also known to modulate Cdc25C. We next determined the levels of Cdc25C by western blotting and found that irradiation increased the levels of Cdc25C protein levels when compared to non-irradiated cells. This increase was further enhanced by SPARC overexpression, thereby suggesting that SPARC overexpression in neuroblastoma cells abates cell cycle arrest and leads to decreased proliferation. Cyclin B is known to be one of the regulatory proteins involved in mitosis and forms a complex with Cdc2. Here, we sought to determine the levels of these proteins by western blotting. Our results demonstrated that Cyclin B and Cdc2 levels were increased in the combination treatment (Fig. 2B), indicating that irradiation-induced G2/M cell cycle arrest was abating by SPARC overexpression in neuroblastoma cells.

### SPARC overexpression decreases radiation-induced PI3K-AKT and PTEN signaling

Ionizing or ultraviolet radiation-induced cellular survival signaling pathways induce development of cancer and insensitivity of tumor cells to radiation therapy [31]. Collecting evidence suggests that the phosphatidylinositide 3-kinase (PI3K)/AKT signal pathway is an important contributor to radioresistance [31]. In many cell types, PI3K/AKT signaling is a key cytoprotective response downstream of the EGFR family receptors and mediates carcinogenesis [31]. The phosphatase and tensin homologue (PTEN) is also a negative regulator of proliferation in many cancer types. Furthermore, AKT activity is elevated in cell lines with the mutated PTEN tumor suppressor gene. Therefore, we sought to characterize the effects of physiologic and genetic manipulation of AKT signaling on combined treatments of IR and SPARC overexpression on neuroblastoma cell proliferation. We first assessed the expression levels of EGFR and PI3K/AKT signaling molecules in the combination treatment. Radiation-induced EGFR phosphorylation and PI3K/AKT levels were inhibited and PTEN levels were increased by SPARC overexpression prior to irradiation in neuroblastoma cells (Fig. 3A). SPARC overexpression prior to irradiation decreased pAKT levels by 60–70% when compared to mock or empty vector-treated controls (Fig. 3B); PTEN levels were increased up to 3- to 4-fold in SPARC-overexpressed neuroblastoma cells when compared to mock or empty vector-treated cells (Fig. 3B) as determined by densitometry analysis.

**Figure 3:** SPARC overexpression inhibits AKT phosphorylation and induces PTEN. SK-N-AS, NB1691 and IMR-32 cells were transfected with mock (PBS control), empty vector (pEV) or with pSPARC for 24 hours, and SK-N-AS and NB1691cells were irradiated (IR) with 8 Gy and IMR-32 cells were irradiated with 4 Gy dose of radiation for further 16 hours. (**A**) Cell lysates were assessed for EGFR, AKT and their phosphorylations, PI3K, mTOR, PTEN and c-Myc by western blotting. (**B**) Protein levels were quantified by densitometric analysis for pAKT and PTEN is shown in the corresponding bar graph. Columns, mean of triplicate experiments; bars, SD. Results are representative of three independent experiments. * *p*<0.01 vs pEV; ** *p*<0.01 vs IR+pEV.

PTEN is capable of modulating the c-Myc gene and has been implicated in the control of cell proliferation, differentiation, and pathogenesis of malignant diseases. We next determined the levels of c-Myc in the combination treatment and observed that c-Myc levels were inhibited by SPARC overexpression, thereby indicating a role of PI3K/AKT signaling in neuroblastoma cell proliferation. AKT has been shown to play an important role in several cellular functions such as cell survival, growth, proliferation, migration, metabolism and angiogenesis [32]. It is clear that AKT has the capacity to act on the substrates affecting various cellular signaling pathways and it was of interest to us to check the role of AKT overexpression in the SPARC-mediated effect of neuroblastoma cell proliferation. To confirm the role of PI3K/AKT pathway in SPARC-overexpressed neuroblastoma cell proliferation, studies were performed using myristoylated (constitutively active) AKT (myr-AKT) overexpression. Earlier reports showed that decreased Chk1 can inhibit the G2 cell cycle arrest [33]. Therefore, we first determined the levels of Chk1 in AKT overexpressed pSPARC-transfected neuroblastoma cells. Activation of AKT signaling by myr-AKT in the SPARC-overexpressed neuroblastoma cells led to decreased cell cycle check point Chk1 (Fig. 4A). In parallel, activation of AKT inhibits SPARC-induced PTEN in neuroblastoma cells (Fig. 4A). To confirm the role of collective inhibition of Chk1 and PTEN on proliferation, we assessed the proliferation rate using MTT assay in AKT overexpressed, pSPARC-transfected cells with or without radiation. The results clearly demonstrate that overexpression of constitutively active AKT led to increased proliferation in irradiated and non-irradiated cells with pSPARC transfection (Fig. 4B).

**Figure 4:** Constitutively active AKT overexpression blocks the radiosensitization capability of SPARC in neuroblastoma cells. SK-N-AS, NB1691 and IMR-32 cells were transfected with mock (PBS control), empty vector (pEV) or with pSPARC alone or in combination with plasmid overexpressing constitutively active AKT (myrAKT; pAKT) for 24 hours, and SK-N-AS and NB1691cells were irradiated with 8 Gy and IMR-32 cells were irradiated with 4 Gy dose of radiation and incubated for further 16 hours. (**A**) Cell lysates were assessed for SPARC, pAKT, EGFR, pEGFR, PTEN, c-Myc and Chk1 by western blotting. Protein levels were quantified by densitometric analysis and shown in the corresponding bar graph. Columns, mean of triplicate experiments; bars, SE. Results are representative of three independent experiments. (**B**) At the indicated time points, the plates were incubated by adding MTT reagent for a further 6 hours. The developed purple color formazan crystals were solubilized using DMSO, and color intensity was measured by spectrophotometer at 570 nm. Data are plotted at an absorbance of 570 nm. Results are representative of three independent experiments. Points, mean of triplicate experiments. H = hours.

### SPARC overexpression induces c-Jun activation and leads to increased PTEN

In certain cancers SPARC is known to increase the levels and activity of the transcription factor c-Jun [34]. We sought to determine the levels of JNK activation as this can potentiate transcriptional activity of c-Jun by phosphorylating serines 63 and 73 [35]. Western blot analysis revealed that SPARC overexpression increased the phosphorylation of JNK by about 2–3 fold in all the cell lines when compared with mock or empty vector-treated neuroblastoma cells (Fig. 5). We evaluated the levels of phosphorylation of c-Jun at serine 63 and 73 upon SPARC overexpression. SPARC overexpression led to increased p-c-Jun (Ser-63) and p-c-Jun (Ser-73) when compared to mock and empty vector-transfected cells (Fig. 5). As JNK is a known modulator of PTEN [36], we further tested whether inhibition of JNK activation will suppress PTEN in neuroblastoma cells. We found that inhibition of JNK using the JNK activation inhibitor reduced the level of PTEN in SPARC overexpressed cells when compared with non-treated SPARC overexpressed neuroblastoma cells (Fig. 5).

**Figure 5:** SPARC overexpression activates JNK and JNK in turn activates PTEN. SK-N-AS, NB1691 and IMR-32 cells were transfected for 24 hours with mock (PBS control), empty vector (pEV) or with pSPARC and treated with or without JNK activation inhibitor (JNK-I) for another 12 hours. Cell lysates were assessed for pJNK, JNK, c-Jun, p-c-Jun (ser-63), p-c-Jun (ser-73) and PTEN by western blotting. Protein levels were quantified by densitometric analysis and shown in the corresponding bar graph. Columns, mean of triplicate experiments; bars, SE. Results are representative of three independent experiments. * *p*<0.01 vs pEV; ** *p*<0.01 vs pEV+JNK-I.

### PTEN overexpression inhibits proliferation in SPARC-inhibited neuroblastoma cells

Direct inhibition of signaling pathways that are negatively regulated by PTEN suppress proliferation and migration in SPARC-expressing GBM cells *in vitro* [37]. PTEN is a negative regulator of AKT that is often mutated or deleted in AIPC, resulting in AKT-mediated survival signaling, which confers chemotherapeutic resistance in AIPC [38]. To examine the effect of PTEN on the phosphorylation status of AKT cell survival signaling pathway, we overexpressed PTEN in SPARC-inhibited neuroblastoma cells. The neuroblastoma cells (SK-N-AS, NB-1691 and IMR-32) were transfected with either SPARC siRNA or with non-specific siRNA for 24 hours, and then treated with PTEN-overexpressing plasmid for a further 24 hours. The results suggested a significant reduction of phosphorylated AKT in SPARC-inhibited neuroblastoma cell lines when PTEN was overexpressed, suggesting that PTEN plays an important role in inhibition of proliferation with the combination treatment (Fig. 6A). MTT assay of the PTEN-overexpressed neuroblastoma cells showed decreased proliferation at the 72-hour time point in SPARC-inhibited cells to 70%, 62% and 75% in SK-N-AS, NB1691 and IMR-32 cells, respectively (Fig. 6B)

**Figure 6:** PTEN overexpression inhibits neuroblastoma cell proliferation in SPARC-inhibited cells. SK-N-AS, NB1691 and IMR-32 cells were transfected with mock (PBS control), empty vector (pEV) or with siRNA against SPARC (pSP-siRNA) alone or in combination with plasmid overexpressing PTEN (pPTEN) for 24 hours. SK-N-AS and NB1691cells were irradiated (IR) with 8 Gy and IMR-32 cells were irradiated with 4 Gy dose of radiation. (**A**) Cell lysates were assessed for SPARC, pAKT, PTEN, c-Myc and Chk1 by western blotting. (**B**) SK-N-AS, NB-1691 and IMR-32 cells were transfected and irradiated as above, and at the indicated time points, the plates were incubated by adding MTT reagent for a further 6 hours. The developed purple color formazan crystals were solubilized using DMSO, and color intensity was measured using a spectrophotometer. Data are plotted as absorbance at 570 nm. Results are representative of three independent experiments. Points, mean of triplicate experiments. H = hours.

### SPARC overexpression inhibits *in vivo* growth capacity of neuroblastoma cells in SCID mice

To assess the effect of SPARC overexpression on sensitizing tumors to radiotherapy, NB1691 neuroblastoma cells were orthotopically injected into the right adrenal gland of SCID mice. After one week of treatments, tumors were removed and fixed in 10% phosphate-buffered formaldehyde. Significant reduction in tumor growth was observed in mice treated with SPARC alone or with SPARC in combination with radiation as compare to mice treated with controls with or without radiation (Fig. 7A). H&E staining for tumor sections showed decreased tumor volume in SPARC-overexpressed mice when compared to mock or empty vector-treated mice with or without radiation (Fig. 7B). To determine SPARC overexpression *in vivo*, tumor sections were stained with a monoclonal antibody for human SPARC. Figure 7C indicates that tumor sections from pSPARC alone or in combination with radiation treatment showed intense staining for SPARC as compared to radiation alone or in combination with mock or the pEV treatment. To assess whether reduced tumor growth was due to inhibition of tumor cell proliferation, we analyzed the levels of Ki67 in the tumor sections. Ki67 staining was found to be higher in mock or pEV treatment alone or in combination with radiation as compared to SPARC treatment alone or in combination with radiation, thereby indicating that SPARC overexpression in *in vivo* reduced tumor cell proliferation (Fig. 7C). To determine whether inhibited proliferation in SPARC-overexpressed tumors was due to decreased AKT and increased PTEN levels, we analyzed AKT and PTEN levels in these tumor sections using specific antibodies against pAKT and PTEN. Tumor sections from either SPARC alone or in combination with radiation showed moderate staining for pAKT. In contrast, we found intense staining for PTEN when compared to mock or pEV treatment alone or in combination with radiation (Fig. 7C). These results are consistent with a role for AKT-PTEN in SPARC-mediated inhibition of proliferation as observed *in vitro*.

**Figure 7:** SPARC overexpression alone and in combination with radiation inhibits neuroblastoma cell proliferation *in vivo* through increased expression of PTEN and inhibited phosphorylation of AKT. Neuroblastoma orthotopic tumor sections from mice injected with mock, pEV or pSPARC plasmids alone or in combination with radiation (IR) were analyzed as described in Materials and Methods. (**A**) Tumor photographs from representing mice, (**B**) Hematoxylin and Eosin (H&E) staining for the tumors (Magnification at 4× and 40×), and (**C**) immunohistochemical analysis for SPARC, Ki-67, pAKT and PTEN were carried out as described in Materials and Methods. All results are representative of multiple tumors taken from five separate mice in each treatment group (Magnification at 60×).

## Discussion

Earlier reports suggested that SPARC negatively regulates cell proliferation in several cancers without stimulating metastasis [39]. In certain cancers, such as melanomas and gliomas, SPARC is associated with a highly aggressive tumor phenotype. In other cancers, mainly ovarian, neuroblastoma, and colorectal, SPARC may function as a tumor suppressor [9]. These opposing effects on cell growth, cell migration and tumor formation suggest that the functions of SPARC are cell-specific and may be dependent upon concentration as well as regulation of ECM components.

Earlier studies [40] were done to investigate the effects of downregulated SPARC expression on the radiosensitivity of human glioma U-87MG cells and its possible mechanism. With a small-interfering RNA (siRNA) expression plasmid vector targeting SPARC, these authors obtained the stably transfected cells in which the expression of SPARC was successfully downregulated. The cells were then irradiated and analyzed by several methods, including clonogenic assay, flow cytometry, comet assay, and western blotting. Clonogenic assay showed that downregulation of SPARC expression enhanced cell survival after radiation. Flow cytometry analysis indicated that SPARC siRNA decreased cell apoptosis responding to irradiation. Analysis of signaling molecules with western blotting showed that the level of AKT phosphorylation was increased in irradiated U-87MG/SPARCsiRNA cells. Further, cell-cycle analysis by flow cytometry showed enhanced G2 accumulation in U-87MG/SPARCsiRNA cells after irradiation. The data suggest that inhibition of SPARC expression may diminish the radiosensitivity of human glioma U-87MG cells. One of the mechanisms for this effect may be associated with the reduced cell apoptosis responding to radiation, which may be contributed by the phosphoinositide 3-kinase/AKT pathway activation. Moreover, the authors hypothesized that enhanced G2 accumulation and increased DNA repair may also account for the decreased radiosensitivity. SPARC is also known for sensitizing therapy-resistant tumors for either chemotherapy or radiation.

Neuroblastoma is the most common pediatric solid tumor. This aggressive embryonal malignancy of neural crest origin has a peak age of onset of 22 months, and accounts for ∼11% of all pediatric cancers and 15% of all pediatric cancer deaths. With current treatment protocols, including chemotherapy, stem cell transplantation, radiation, and surgery, ∼80% of high-risk patients go into remission, although the majority relapse and succumb to therapy-resistant tumors.

The role of SPARC in cell survival and death is complex. SPARC was originally identified as a stress response gene [41] and subsequently described as a c-Jun-responsive target gene that can be repressed or induced depending on cell type [42], [43]. On the other hand, there is evidence in some contexts that SPARC induces apoptosis in ovarian cancer cells [44] and modulates sensitivity to chemotherapy in colon cancer cells by enhancing apoptosis [45]. Therefore, the focus of this investigation was to determine the role of SPARC in neuroblastoma cell proliferation. Our earlier findings revealed that proliferation, adhesion, migration, invasion, and MMP-9 activity in medulloblastoma (data published earlier) [12], could be inhibited by SPARC. We have also shown in an earlier study that SPARC induced autophagy-mediated apoptosis in PNET tumor cells [12]. Here, we sought to determine the mechanism by which SPARC could inhibit neuroblastoma cell proliferation. Moreover, SPARC overexpression increased the levels of tumor suppressor protein PTEN and inhibited pro-proliferating protein AKT. These results demonstrate that SPARC has the potential to inhibit neuroblastoma cell proliferation, thereby leading to reduced tumor growth.

In the present study, we used a plasmid encoding the SPARC full-length gene for SPARC overexpression in the neuroblastoma cell lines to determine proliferation rate and tumor growth. The cells transfected with pSPARC showed a 3- to 4-fold increase in protein levels (as determined by western blotting and immunocytochemical analysis) and in gene transcript levels (as determined by RT-PCR analysis) when compared to mock or empty vector-transfected cells. SPARC overexpression inhibited neuroblastoma cell proliferation as determined by MTT assay.

Previously, SPARC was shown to be an anticipated resistance-reversal gene as evidenced by low SPARC expression in refractory human MIP101 colon cancer cells [24]. Restoration of cells radiosensitivity and chemosensitivity was achieved by re-expression of SPARC in tumor xenografts of colon cancer. Additionally, mice treated with SPARC showed increased sensitivity to chemotherapy, which led to significant regression of xenografted tumors. Earlier reports showed that modulation of SPARC expression affected colorectal cancer sensitivity to radiation and chemotherapy [24]. In the present study, SPARC expression levels were reduced with radiation in a dose-dependent manner in neuroblastoma cell lines. SK-N-AS and NB1691 cells showed radiation resistance until 8 Gy radiation, whereas IMR-32 cells showed resistance only until 4 Gy. It is well known that when cells are exposed to radiation, they cause a complex response that includes cell cycle arrest in G1 and G2 phases [26], [46]. DNA is an important subcellular target of ionizing radiation, but oxidative damage to plasma membrane lipids initiates signal transduction pathways that activate apoptosis, which may play a role in cell cycle regulation [47]. In this study, we illustrate that SPARC alters the cell cycle and sensitizes neuroblastoma cells to radiation by altering Chk1 and Cdc25C. Earlier reports [48] show that cyclin B increase can also occur in the absence of spindle inhibition if c-Myc deregulation is combined with inactivation of the p53 tumor suppressor. Under these conditions, cyclin B1 protein is induced but retains its normal cell cycle regulation. The authors show that c-Myc and the loss of p53 cooperate to induce cyclin B1 mRNA and protein. The central role of cyclin B1 in the maintenance of genomic integrity is underscored by the consequences of its deregulated expression. This may be one of the reasons for the increase in the cyclin B levels in the SPARC treatment

MAPK families are known to play an important role in key cellular processes including proliferation, differentiation, development, transformation, and apoptosis [49]. We evaluated the levels of JNK in SPARC-overexpressed neuroblastoma cells and found increased activation of JNK. Earlier reports showed that the treatment of the colon cancer cell line HT29 with the differentiating agent sodium butyrate (NaBT) increased PTEN protein and mRNA expression and also induced c-Jun NH2-terminal kinase (JNK) activation. Inhibition of JNK by chemical or genetic methods attenuated NaBT-induced PTEN expression [36]. We observed that SPARC overexpression increased the activation of JNK and led to increased PTEN levels which were inhibited by the JNK specific inhibitor. Based on the these results, we hypothesize that SPARC activates JNK and activated JNK leads to increased PTEN levels in SPARC-overexpressed neuroblastoma cells.

SPARC overexpression in neuroblastoma cells prior to radiation inhibited AKT phosphorylation and increased levels of the PTEN tumor suppressor protein. Accumulating evidence suggests that the phosphatidylinositide 3-kinase (PI3K)/AKT signal pathway is a major contributor to radioresistance [31]. Earlier reports suggested that activation of the PI3K/AKT pathway is also associated with tumorigenesis and resistance to apoptosis [50], [51]. To confirm the role of the AKT pathway in sensitizing SPARC capabilities towards radiation in neuroblastoma, we overexpressed activated AKT using myr-AKT. The results suggest that activation of AKT in the presence of SPARC overexpression led to increased proliferation in neuroblastoma cells prior to radiation. We further determined that phosphorylation of EGFR was inhibited with SPARC overexpression prior to radiation in these cells. In many cell types, PI3K/AKT signaling is a key response downstream of the EGFR family of receptors and mediates carcinogenesis [31].

Moreover, AKT activity is commonly dysregulated in a variety of human tumors because of frequent inactivation of the PTEN tumor suppressor gene, which negatively regulates phosphatidylinositol 3 phosphate levels [52], [53]. Moreover, alterations of this gene have been identified in a large fraction of cancers [36], [54], [55]. In light of this, we postulate that increased PTEN function with subsequent inhibition of SPARC prior to radiation reduced AKT phosphorylation, thereby leading to decreased proliferation in neuroblastoma cells. PTEN reduced AKT signaling in both control and SPARC-overexpressing cells, suggesting that PTEN signaling works as a downstream effector for SPARC overexpression in neuroblastoma cells. In the current study, we found that SPARC overexpression increased PTEN levels both *in vitro* and *in vivo*. One possible explanation is that when PTEN is expressed, the resulting suppression in cell growth may induce the cells to become more dependent on growth factor signaling, which can be antagonized by SPARC.

Our *in vitro* data indicated that SPARC inhibited proliferation and sensitized neuroblastoma cells to radiation via reducing the phosphorylation levels of AKT, thereby leading to increased PTEN. Moreover, our *in vitro* data also showed that both SPARC and PTEN were expressed at the same time and followed inhibition of pAKT in tumor cells when treated with pSPARC. We expected the same results *in vivo*. To test this hypothesis, we orthotopically grafted mice with NB1691 neuroblastoma cells and treated them with mock, pEV or pSPARC alone or in combination with radiation. The animals treated with pSPARC showed increased SPARC levels as compared to mock or empty vector-treated tumors. Immunohistochemical analysis for PTEN and pAKT demonstrated that SPARC and PTEN were overexpressed when treated with pSPARC and at the same time, pAKT was inhibited, leading to reduced proliferation *in vivo*. Other studies support our findings since SPARC-overexpressing glioma cells have been reported to inhibit cell proliferation upon PTEN induction [37]. Accordingly, the addition of SPARC was shown to modulate the proliferation of many primary cells including endothelial cells [56], [57], skeletal myoblasts [58], mesangial cells [59], mesenchymal cells [60], mesothelial cells [44], and epithelial cells [61]. The effect that changes in SPARC levels have on tumor cell proliferation is more complex and debatable.

Earlier studies [62] showed that SPARC expression is inversely correlated with the degree of malignant progression in neuroblastoma tumors. Knockdown of SPARC in neuroblastoma cells may increase the malignant progression in neuroblastoma tumors. SPARC has also been shown to have a role in growth rate modulation as demonstrated by SPARC knockout mice having an increased rate of tumor growth than those mice with intact SPARC [63], [64]. Based on the literature available, it may be possible that forced knockdown of SPARC in these conditions may lead to more tumor growth. Said and Motamed [65] evaluated the effect of host-derived SPARC on ovarian cancer growth *in vivo*, demonstrating more rapid and aggressive tumor growth in SPARC-deficient animals.

In summary, we have shown that overexpression of SPARC decreases proliferation and sensitizes neuroblastoma cells to irradiation. We hypothesized that overexpression of SPARC resulted in inhibition of pAKT and increased PTEN, leading to cell cycle abate that subsequently caused the inhibition of proliferation and sensitized cells to radiation *in vitro* and *in vivo*. On the basis of these observations, we conclude that endogenous overexpression of SPARC can decrease neuroblastoma cell proliferation and tumor growth and therefore act as a tumor suppressor in human neuroblastoma. Future studies in human neuroblastoma should focus on the design of treatment strategies that specifically target SPARC–PTEN interactions.

## Materials and Methods

### Ethics statement

The Institutional Animal Care and Use Committee of the University of Illinois College of Medicine at Peoria, Peoria, IL, USA, approved all surgical interventions and post-operative care. The consent was written and approved. The animal protocol number is 872, dated May 20^th^ 2010 and renewed on May 20^th^ 2011.

### Cell culture

SK-N-AS and IMR-32 cells were obtained from ATCC (Manassas, VA) and NB-1691 cells were obtained from Dr. Houghton of St. Jude Children's Research Hospital (Memphis, TN). Cells were cultured in RPMI medium with 10% fetal bovine serum, 2 mM/L L-glutamine, 100 units/mL penicillin, and 100 µg/mL streptomycin. Cells were maintained in a humidified atmosphere containing 5% CO2 at 37°C.

### Antibodies and reagents

Antibodies against SPARC, pAKT, AKT, c-Myc, PTEN, EGFR, pEGFR, Cyclin B, Cyclin D1, Cdc2, pCdc2, Cdc25C, Chk1, Chk2, mTOR, PI3K, JNK, pJNK, c-Jun, p-c-Jun (Ser-63), p-c-Jun (Ser-73), caspase-3, and GAPDH were obtained from Santa Cruz Biotechnology (Santa Cruz, CA), Antibodies against PARP (Cell Signaling Technology, Beverly, MA) were also used in this study. Plasmids encoding myr-AKT delta4–129 (Addgene plasmid 10841) and HA PTEN wt (Addgene plasmid 10750) were obtained from Addgene Inc. (Cambridge, MA).

### Construction of pcDNA3.1-SPARC and transfection

An 1100-bp cDNA fragment of human SPARC was amplified by PCR using synthetic primers and sub-cloned into a pcDNA3.1 vector (Invitrogen, San Diego, CA) in the “sense” orientation. Neuroblastoma cells were transfected with full-length cDNA SPARC-containing vector using FuGene HD (Roche, Indianapolis, IN) as per the manufacturer's protocol.

### siRNA design and transient transfection

SPARC siRNA sequences were designed with the help of a siRNA designer program (Imgenex, Sorrento Valley, CA). The siRNA was complementary to an exonic sequence of the target mRNA and compatible with the pcDNA3.1 vector (Invitrogen, San Diego, CA). The following siRNA sequence was used to construct SPARC siRNA and designated as SP-siRNA: 5′-TCGAGGGTGTGCAGCAATGACAA CAAGAGTCGTCGTTGTTGTCATTGCTGCACACCG-3′. A control vector containing siRNA with a scrambled sequence was constructed and designated as control siRNA. We used the following scrambled sequence: 5′-CACGGAGGTTGCAAAGAATAATCGATTATTCTTT GCAACCTCC GTGC-3′.

### Transfection with plasmids

All transfection experiments were performed using FuGene HD transfection reagent according to the manufacturer's protocol (Roche). Briefly, plasmid/siRNA was mixed with FuGene HD reagent (1∶3 ratio) in 500 µL of serum-free medium and left for 30 min to allow for complex formation. The complex was then added to the 100-mm plate, which had 2.5 mL of serum-free medium (2 µg plasmid per ml of medium). After 6 hours of transfection, complete medium was added and cells were cultured for another 36 hours.

### Immunocytochemistry

We used a previously described protocol with minor changes [66]. Briefly, the cells were cultured on 8-well chamber slides and fixed with 4% paraformaldehyde (w/v) in PBS, permeabilized with 0.1% Triton X-100 (w/v) in PBS and blocked with 1% BSA (w/v) in PBS for 1 hour at 4°C. Cells were incubated overnight at 4°C with anti-SPARC antibody followed by corresponding Alexa fluor-594-conjugated secondary antibody for 1 hour and counterstained with DAPI. For negative controls primary antibody was replaced by non-specific IgG. Slides were washed and mounted with anti-fade mounting solution (Invitrogen, San Diego, CA) and analyzed with an inverted microscope.

### Western blotting

Western blot analysis was performed as described previously [67]. Briefly, 36 hours after transfection, cells were collected and lysed in RIPA buffer. Equal amounts of protein were resolved on SDS-PAGE and transferred onto a PVDF membrane. The blot was blocked with 5% non-fat dry milk and probed overnight with primary antibodies followed by HRP-conjugated secondary antibodies. An ECL system was used to detect chemiluminescent signals. All blots were re-probed with GAPDH antibody to confirm equal loading.

### RT-PCR

Neuroblastoma cells were transfected with mock, pEV or pSPARC for 36 hours. Total RNA was extracted from these cells and cDNA synthesized using poly-dT primers as described earlier [68]. PCR was performed using the following primers: SPARC: 5′-GGAAGAAACTGTGGCAGAGG-3′ (sense), and 5′-ATTGCTGCACACCTTCTCAA-3′ (antisense); GAPDH: 5′-TGAAGGTCGGAGTCAACGGATTTGGT-3′ (sense), and 5′-CATGTGGGCCATGAGGTCCACCAC-3′ (antisense). Quantification of SPARC mRNA levels was determined based on densitometry.

### Flow cytometry

For assessment of DNA content, neuroblastoma cells were plated overnight in 100-mm tissue culture plates and transfected for 36 hours as described above. We used FACS analysis that utilizes propidium iodide staining of nuclear DNA to characterize hypo-diploid cells [69]. Briefly, cells were harvested by trypsinization and stained with propidium iodide (2 mg/mL) in 4 mM sodium citrate containing 3% (w/v) Triton X-100 and RNase A (0.1 mg/mL; Sigma, St. Louis, MO). Suspensions of 2×10^6^ cells were analyzed by FACS Caliber System (Becton Dickinson Bioscience, San Jose, CA) with laser excitation at 488 nm and using an emission 639 nm band pass filter to collect the red propidium iodide fluorescence. The percentages of cells in the various phases of the cell cycle (sub-G1, G1/S, and G2/M) were assessed using Cell Quest software (Becton Dickinson Bioscience).

### Cell proliferation assays

Cell growth rate was determined using a modified 3-(4,5-dimethylthiazol-2-yl)-2,5-diphenyltetrazolium bromide (MTT) assay as a measurement of mitochondrial metabolic activity as described earlier [70]. Cells were transfected with indicated plasmids and incubated at 37°C. After 0 to 72 hours, MTT reagent was added to the cells and incubated for 6 hours at 37°C. The rate of absorbance of formazan (a dye produced by live cells) was measured with a microplate reader at A550.

### Clonogenic assay

Cells were transfected with mock, pEV, and pSPARC for 24 hours and irradiated with different Gy of radiation. Cells (5×10^2^ cells) were trypsinized and seeded in 100 mm Petri dishes. On day 10 after irradiation, cells were fixed in cold methanol and stained with Giemsa and colonies (>50 cells) were counted. The plating efficiency (PE) is defined as the number of colonies observed/the number of cells plated. Surviving fraction (SF) is the colonies counted divided by the number of colonies plated with a correction for the plating efficiency.


### Intra-adrenal tumor model and immunohistochemistry

The Institutional Animal Care and Use Committee at the University of Illinois College of Medicine at Peoria approved all experimental procedures involving the use of animals. Orthotopic, localized neuroblastoma tumors were established in C.B-17 SCID mice by injection of 1×10^6^ NB-1691 cells in 100 µL PBS into the retroperitoneal space as described earlier [71]. After 2 weeks of tumor cell implantation, the mice were separated into six groups containing 6 animals per group, and each group was injected intravenously with PBS (mock) or pEV or pSPARC (100 µL volume) and was given three doses on alternate days. Between the first and the second injections, and the second and the third injections, one group was radiated with a dose of 5 Gy each time. Mice were euthanized when animals had lost >20% of body weight or had trouble ambulating, feeding, or grooming. The tumors were removed and either fixed in 10% phosphate-buffered formaldehyde or snap frozen and maintained at −70°C until sectioning. Briefly, all tumors were serially sectioned and tissue sections (7 µm thick) obtained from the paraffin blocks were stained with hematoxylin and eosin (H&E) using standard histologic techniques. For immunohistochemical analysis, sections were incubated with mAb (1 hour at room temperature) followed by the appropriate secondary antibody. For HRP-conjugated secondary antibodies, we used DAB solution as the chromogen. Negative control slides were obtained by nonspecific IgG. Sections were mounted with mounting solution and analyzed with an inverted microscope.

### Statistical analysis

All data are expressed as mean ± SD. Statistical analysis was performed using the student's *t* test or a one-way analysis of variance (ANOVA). A *p* value of less than 0.05 was considered statistically significant. All experiments were performed in triplicate to obtain consistent results.

## Supporting Information

Figure S1 **Overexpression of SPARC in neuroblastoma cells.** The human full-length SPARC cDNA was subcloned into the pDNR-CMV mammalian expression vector and termed as pSPARC. pDNR-CMV was the vector without the SPARC gene and termed as empty vector (pEV). SK-N-AS, NB1691 and IMR-32 cells were transfected with mock (PBS control), empty vector (pEV) or SPARC full-length gene inserted vector (pSPARC) for 36 hours. (**A**) SPARC levels were determined by Western blotting using a SPARC-specific antibody. GAPDH served as a loading control. Columns, mean of three experiments; bars, SD.* *p*<0.01 vs pEV. (**B**) cDNA was produced from total RNA extracted from the mock and infected cells. RT-PCR analysis was performed for SPARC. Results are representative of three independent experiments. GAPDH served as a control for RNA quality. Columns, mean of three experiments; bars, SD. * *p*<0.01 vs pEV. (**C**) SK-N-AS, NB1691 and IMR-32 cells were transfected with mock (PBS control), empty vector (pEV) or pSPARC for 36 hours and immunocytochemical analysis for SPARC was performed. Representing images were shown taken from 5 different microscopic fields of three independent experiments. (**D**) SK-N-AS, NB1691 neuroblastoma cells and HMEC cells were culture for 24 hours and Western blot analysis was performed for SPARC using specific antibody. GAPDH served as loading control. (**E**) Clonogenic survival assay for irradiated neuroblastoma cells. SK-N-AS, NB1691 and IMR-32 neuroblastoma cells were irradiated (IR) with 2 Gy to 12 Gy doses of radiation and clonogenic assay was performed as described in Materials and Methods. The cells were culture and colonies larger than 50 cells were counted. Points: mean of triplicate experiments.
(TIF)
